# Protective effect of crocin-loaded nanoparticles in rats following epileptic seizures: Biochemical, behavioral and histopathological outcomes

**DOI:** 10.1016/j.heliyon.2024.e36122

**Published:** 2024-08-10

**Authors:** Cyrus Jalili, Mohammadreza Gholami, Seyran Kakebaraei

**Affiliations:** a Medical Biology Research Center, Health Technology Institute, Kermanshah University of Medical Sciences, Kermanshah, Iran; b Department of Anatomical Sciences, Kermanshah University of Medical Sciences, Kermanshah, Iran; c Anatomy Students Research Committee, Kermanshah University of Medical Sciences, Kermanshah, Iran

**Keywords:** Epileptic seizures, Crocin, Nanotechnology, Oxidative stress, Memory

## Abstract

Epilepsy is a condition resulting from complex interactions involving excessive neuronal electrical activity and oxidative stress, which can lead to chronic neurological conditions. This study evaluates crocin encapsulated in SLNC for neuroprotective and countering pentylenetetrazole (PTZ) -induced oxidative damage. The rats were pre-treated with SLNC and FC (25, 50 mg/kg/day; P.O.) for 28 days before being induced with PTZ. Various standard tests were conducted to assess their behavioral functions, such as Y-maze, Open field test (OFT), and elevated plus maze (EPM) tests. ELISA measured brain tissue catalase activity (CAT) and nitric oxide status (NO). The expression of Nuclear factor kappa B (NF-κB) and the number of dendrite spines were examined through Immunohistochemical and Golgi–Cox staining, respectively. The Pretreating rats with SLNC plus PTZ significantly boosted memory and reduced anxiety levels in Y-maze, OFT, and EPM tests. In addition, it decreased NO levels and increased CAT levels. SLNC also showed a significant decrease in NF-κB expression and an increase in neurons and the number of spines. The positive effects of SLNC in improving memory and learning deficits after PTZ injection can be attributed to its anti-inflammatory and anti-oxidative effects.

## 1 Introduction

Epilepsy comprises a range of non-communicable diseases related to the central nervous system (CNS), distinguished by repeated seizures without fever or toxic-metabolic triggers, as well as cognitive and emotional disturbances [1]. Although there is widespread recognition of the epidemiological aspects of this disorder, there are substantial concerns regarding the nature, timing, and course of the disease, causal relationships, and clinical interventions to prevent progression and manage epileptic patients [2]. Of particular concern is the extent to which chronic, drug-resistant epilepsy may lead to progressive depressive behavior and cognitive deficits [3]. Seizures typically begin with abnormal electrical discharge, which leads to excessive excitation or synchronization of neurons in the CNS. Nevertheless, seizures' exact signs and presentations are relevant to several factors, such as the time of onset, location in the cerebral, and presence of underlying diseases or conditions [4]. Seizures possess the ability to affect motor skills, cognition, and even one's state of consciousness [5]. It should be pointed out that various factors, including oxidative damage, neuroinflammation, uncontrolled release of neurotransmitters, and cell death, cause epilepsy. The hippocampus can become more susceptible to seizures due to the induction of neuroinflammation and oxidative injury [6]. In neonatal and adult animals, acute inflammation can change brain excitability and heightened susceptibility to seizures [7]. Prescribed to alleviate seizures, anti-epileptic drugs (AEDs) work by blocking sodium channels, regulating neurotransmitter release, and modulating synaptic receptors. Unfortunately, around one-third of individuals with epilepsy do not respond to the existing classical AEDs. To make matters worse, these drugs sometimes come with side effects that have the potential to adversely affect quality of life and hinder treatment adherence [8,9]. It is important to continue researching new, safer neuroprotective ingredients with anticonvulsant properties. Medicinal herbs show promise in this field of research. In vivo studies have demonstrated certain plants' antiepileptic and sedative effects, indicating their potential effectiveness in managing seizures. These findings emphasize the potential of traditional herbal medicine as a therapeutic option for individuals with epilepsy (10, 11). Crocin is a main constituent of Crocus sativus L., which has various pharmacological properties such as anti-diabetic, pain-relieving, antioxidant, antitumor, anti-inflammatory, neuroprotective, and anti-apoptotic [10]. Recently, results have been found that safranal has antiepileptic activity in animal models. Furthermore, it has been shown to control seizures induced by maximal electroshock and pentylenetetrazole (PTZ). Also, it exhibits neuroprotective efficacies by exerting antioxidant activity and attenuating cerebral ischemia in rat hippocampus [11]. On the other hand, the blood-brain barrier (BBB) represents a major challenge to drug delivery to the nervous system. The dysfunction of BBB has been reported to play a role in the development of seizures and medication resistance, primarily by limiting the bioavailability of medicines [12]. Thus, nanoparticles (NPs) provide a more precise method of drug delivery for a wide range of therapeutic agents to the brain, overcoming the major obstacle of the BBB. However, nano-antioxidants offer a promising strategy for improving the delivery of antioxidant supplements by addressing the limitations associated with crocin [13,14]. These limitations include inadequate stability, short biological half-life, rapid absorption and metabolism, and poor bioavailability. Nano-drug delivery systems show potential for preventing and treating neurological disorders [14]. Lipid NPs are an efficient method for transferring medicine that mainly distributes into the lipidic matrix of NPs. Solid lipid nanoparticles (SLNs) are the drug carriers of submicron-sized particles (50–1000 nm) created by the blend of liquid and solid lipids. SLNs have distinctive properties, such as high surface area, tiny size, and high drug-carrying capacity, which make them highly promising for delivering pharmaceuticals and nutraceuticals across BBB [13]. Therefore, encapsulation not only improves the brain-targeting abilities of crocin but also has the potential to overcome its quick metabolism and low bioavailability. Hence, the scope of relevant studies was designed to evaluate the beneficial effect of pretreatment of crocin-loaded SLNs (SLNC) in the biochemical, behavioral, and histopathological changes after the administration of PTZ-induced oxidative stress.

## 2 Materials and methods

### 2.1 Animals

Young male Wistar rats (8–12 weeks old; Animal House, Pasteur Institute, Tehran, Iran) weighing 180–200 g were used for the study. The animals were housed in standard laboratory conditions with a 25 ± 2 °C temperature and humidity ranging from 60 % ± 15 %. They were kept on a regular light-dark cycle and had access to food and water at all times. Before the experiment, the animals had grown acclimatized to the laboratory conditions. The experimental protocols received approval from the Ethics Committee of the Kermanshah University of Medical Sciences, Kermanshah, Iran (IR.KUMS.AEC.1401.008).

### 2.2 Chemicals

Crocin (purity ≥98 %, sigma), PTZ, Stearic acid, lecithin, chloroform, Polysorbate 80 (Tween 80), ethylenediaminetetraacetic acid (EDTA), and ethanol are purchased from Sigma-Aldrich (Germany). Anti- NF-κB antibody (cat. no. ab110304) is obtained from Abcam. All other chemicals or solvents used in the research were of analytical grade.

### 2.3 Preparation and characterization of SLNC

Stearic acid, soy lecithin, and pure water were combined and heated in a beaker until reaching the lipid melt temperature (70–75 °C). After introducing crocin into the aqueous phase with Tween 80, the resulting hot emulsifier mixture was swiftly added to the lipid melt, creating a transparent microemulsion. This hot microemulsion was then transferred to cold water (4 °C) and mechanically stirred for 1 h, leading to the formation of SLNC through the crystallization of oil droplets in the microemulsion. Finally, the SLNC was stored in a refrigerator for preservation [15]. The surface and form of the SLNC specimen are examined using Field Emission Scanning Electron Microscopy (FE-SEM) equipment (Zeiss, Sigma VP, Germany). A layer of gold is applied to enhance the SLNC using an ion sputter. Subsequently, photo-micrographs of the SLNC are captured at a suitable magnification. The developed nanoformulation was analyzed using Fourier transform infrared (FT-IR) spectroscopy (FTIR, Shimadzu Co., Japan) to determine its molecular structure accurately.

### 2.4 Calculation of lethal dose of SLNC

The Lethal Dose 50 (LD50) of SLNC is calculated using the oral method on Wistar rats following the Reed and Muench technique [16]. To find the LD50, various doses of SLNC (25, 50, 100, 250, 500, 750, 1000, and 1500 mg/kg) dissolved in normal saline are administered to different groups of rats. From the results of LD50, the provided SLNC concentration is 25 and 50 mg/kg for oral administration. These doses did not cause any adverse effects.

### 2.5 Experimental design

A total of 56 animals were involved in the study, and they were divided into 7 groups through random allocation. The study investigated the protective potential of crocin suspended in 0.9 % NaCl (Free crocin (FC)) and SLNC administered by oral gavage against PTZ. The groups were as follows: Group I – naïve control operated rats (control/0.9 % NaCl); Group II – rats subjected to PTZ (PTZ Control); Group III – rats receiving Blank-SLNs (50 mg/kg-PTZ); Groups IV and V – rats receiving SLNC (25 and 50 mg/kg plus PTZ, respectively); Group VI and VII – rats receiving FC (25 mg/kg and 50 mg/kg plus PTZ, respectively). After 4 weeks of pretreatment with SLNC, FC, and saline administration, epileptic seizures were induced by intraperitoneal (IP) injection of PTZ at a dose of 75 mg/kg [17]. We conducted a comprehensive set of behavioral, biochemical, and histopathological studies on animal groups that were assigned randomly.

### 2.6 Behavioral and biochemical assessment

#### 2.6.1 Seizure severity score

Animals behavior was noticed for 40 min immediately after PTZ administration, and a seizure index score was then determined using the modified Racine scale: 0 = no behavioral change, 1 = whisker tremor, 2 = facial muscle contraction, 3 = Facial jerking, 3 = neck twitching, 4 = clonic seizure onset, 5 = dorsal collapse and tonic-clonic seizure, 6 = death. The duration of the seizures was also recorded [18].

#### 2.6.2 Y-maze test

We evaluated spatial working memory 24 h after PTZ administration using a Y-maze, following the method outlined by Dellu et al. The Y-maze used in the study consisted of three arms crossing at 120° angles, each measuring 35 cm in length, 8 cm in width, and 15 cm in height. Each rat was placed in the maze's center and allowed to explore for 5 min, with the number and sequence of arm entries being recorded. An actual alternation was considered to occur when consecutive entries were made into all three arms (i.e., ABC, BCA, CAB, but not ABA). To calculate the final scores, we have utilized a formula that involves (actual alternation/maximal alternation − 2) × 100 [19].

#### 2.6.3 Elevated plus maze (EPM) test

The elevated plus-maze (EPM) is a widely used tool for evaluating anxiety in laboratory model animals. This device is composed of two open arms measuring (40 cm × 10 cm × 1 cm), and two enclosed arms measuring (40 cm × 10 cm × 40 cm). They are separated by a central support at a height of 50 cm from the floor. At the start of the experiment, the animal is placed in the center of the EPM, facing a closed arm, and allowed to freely explore the maze for 5 min. The rats' behavior during the experimental sessions (5 min) is recorded 48 h after the PTZ injection by a camera positioned above the maze. The recorded behavior is then analyzed for conventional anxiety indicators, including (1) the total distance covered by the animals, (2) the time spent in open arms, and (3) the number of entries into open arms during the test session [20].

#### 2.6.4 Open-field test (OFT)

The open field test (OFT) was used to examine anxiety-related behavior and to detect changes on the 31st day after drug treatment [21]. Pretreated and control epileptic rats were placed in the center of a black square (27 × 27 × 20.3 cm) to freely prospect the district, and their activity was monitored for 15 min (video system Med Associates, USA) in terms of mean speed and distance traveled recorded.

#### 2.6.5 Assessment of griess assay and catalase activity (CAT)

Nitrite oxide (NO) was assessed by Griess assay. In this process, we centrifuged homogenized brain tissue at 3000 rpm for 15 min, and then zinc sulfate (6 mg) was added to the supernatant (400 μL), and centrifuged (4 °C, 12,000 rpm). Briefly, after adding 100 μl of Griess reagent (Sigma; USA) to the samples, the reaction mixture was incubated at room temperature. The absorbance values were read at 540 nm by ELISA plates [22]. CAT activity in rat brain tissue was evaluated at 240 nm using an ultraviolet–visible spectrophotometer (Shimadzu, Japan) using Aebi's procedure [23].

### 2.7 Golgi-cox staining

To evaluate the effects of SLNC, FC plus PTZ on neural morphology in brain tissue of animals, a modified Golgi–Cox stain method was used [17]. Briefly, the rats were dissected, and their brains were meticulously removed and soaked in a solution (A/B = 1:1, 15 ml/rat) in a dark room at room temperature for 2 weeks. Subsequently, the brains were coronally sliced (100 μm), cleaned with xylene, and cover-slipped with gelatin for light microscopic observation. Spine densities were then assessed using an optical microscope and Motic software (version 3).

### 2.8 Immunohistochemical of nuclear factor kappa B (NF-κB) in brain tissue

The NF-κB expression in rat brain tissue was studied using the avidin–biotin–peroxidase technique in an IHC study. Following deparaffinization and hydration, the tissue sections were incubated in peroxidase solution (H2O2) at room temperature to prevent inaccurate staining, and then with primary anti- NF-κB antibodies (Abcam, MA, USA) for 24 h at 4 °C. After three washes in phosphate-buffered saline (PBS), incubated with a secondary antibody for 30 min. Antibodies were detected with horseradish peroxidase-conjugated streptavidin to rabbit IgG, and finally, 3,30-diaminobenzidine (DAB) was smeared, after that hematoxylin stain was applied for counterstaining. NF-κB expression was assessed by determining the number of NF-κB (+) cells in random tissue sections on every slide.

### 2.9 Statistical analysis

The data was analyzed using GraphPad Prism version 9 software. A one-way analysis of variance (ANOVA) and Tukey posttest were performed for the parameters (biochemical analysis and behavioral tests) to compare responses between groups. Quantitative data were presented as mean ± SD. p-value ≤0.05 was considered statistically significant.

## 3 Result

### 3.1 Characterization of SLNC

The emulsion solvent-evaporation technique was utilized to successfully prepare SLNC in this study. The NPs were assessed for their particle size, shape (FESEM), and long-term stability (see Fig. 1A). The average particle size of the SLNC was 98.25 nm, with a polydispersity (PDI) of 0.11 ± 0.13 and a zeta potential of −33.45 mV, indicating consistent size and stability (see Fig. 1). Peaks at 3381 cm^−1^ for N–H symmetric stretch in lecithin and 1734 cm-1 for C=O of the ester compound in lecithin are indicative of functional groups. Additionally, peaks at 2918 and 2852 cm^−1^ for C–H group stretching suggest the presence of a hydrophilic environment in the surfactant, which contributes to the shielding efficacy. Turning to the FTIR spectra of FC, significant bands at 1635 cm^−1^ for the C=C bond, 1492 cm-1 for the C=O bond, and 2922 cm^−1^ for the C–H bond highlight the key functional groups. Specifically, the peaks at 1492 cm^−1^ and 1041 cm^−1^ can be linked to stretching oscillations of C=O in the carbonyl group and C–O stretching vibration, respectively, in the sugar functional groups of crocin structures. The broad stretches at 3427 and 3419 cm^−1^ correspond to the presence of OH groups. Notably, the FTIR spectrum of SLNC shows the presence of unique bands of OH at 3427 and 3419 cm^−1^, which are exclusive to crocin. This confirms the successful interaction between SLN and crocin, highlighting the strong hydrophobicity character of the samples. Therefore, the characteristic peaks observed between SLN and SLNC are likely due to the hydrogen bond constitution when crocin is incorporated into SLN (see Fig. 1B).

**Fig. 1:** (A) FESEM images of SLNC. The scale bar represents 200 nm. The average diameter is 98 ± 25 nm, and the zeta potential is −33.45 mV. (B). FTIR.

### 3.2 LD50 of SLNC

From the results of LD50, the concentration of the provided SLNC is found to be 25 and 50 mg/kg for the oral administration. These doses did not reason any adverse effects.

### 3.3 SLNC pretreament induces antioxidant effect on PTZ severity score

Administration of PTZ at a dose of 75 mg/kg caused tonic, myoclonic, and generalized seizures, which were evaluated using the Racine scale (see Table 1). As indicated in Table 1, treating animals with SLNC plus PTZ at 25 and 50 mg/kg doses for 28 days consistently decreased seizure activity, like duration, flexion, extension, and clonus. This combination demonstrated anticonvulsant effects when compared to PTZ group. However, administering FC plus PTZ at 25 mg/kg before treatment did not significantly alter seizure indicators compared to PTZ group alone. These findings suggest that the SLNC plus PTZ combination holds promise in managing seizure activity. Further exploration of varied dosages and durations may unveil its full therapeutic potential. (^@, #^p < 0.0001).

**Table 1:** Effects of orally administered SLNC and FC plus PTZ on behavioral changes induced by PTZ in seizure scoring: No. Of Convulsion, Duration of the Seizure, Flexion, Extension, Clonus in min.

Groups	No. of Convulsion	Duration of the Seizure (min)	Flexion (min)	Extension (min)	Clonus (min)
Control	0/8	0.0 ± 0.0	0.0 ± 0.0	0.0 ± 0.0	0.0 ± 0.0
PTZ	8/8	28.88 ± 1.72^a^	9.12 ± 1.12^a^	14.38 ± 0.91^a^	8.75 ± 0.7^a^
Blank + PTZ	8/8	28.50 ± 1.19	8.87 ± 0.83	14.38 ± 1.18	8.75 ± 0.7
SLNC25 mg/kg + PTZ	2/8	5.25 ± 0.7^b^	1.62 ± 0.74^b^	2.75 ± 0.70^b^	2.00 ± 0.53^b^
SLNC50 mg/kg + PTZ	1/8	2.75 ± 0.46^b^	0.62 ± 0.51^b^	0.87 ± 0.83^b^	1.00 ± 0.75^b^
FC25 mg/kg + PTZ	7/8	25.88 ± 2.64	8.12 ± 0.83	13.00 ± 0.75	8.5 ± 0.53
FC50 mg/kg + PTZ	5/8	24 ± 1.6^b^	7.25 ± 0.7^b^	11.63 ± 0.91^b^	7.5 ± 0.75^b^

Note: The letters '@' and '#' denote significant differences compared to the untreated control and PTZ-injected alone groups, respectively.

a P < 0.0001 compared with the control group.

b P < 0.0001 as compared with the PTZ group alone. All data is presented as mean ± standard deviation (SD); n = 8 animals per group.

### 3.4 Y-maze test

The Y-maze test finding revealed a notable decrease in total arm entries and spontaneous alternation behavior in the PTZ group alone compared to the control (****p < 0.0001). Conversely, the groups treated with SLNC at concentrations of 25 and 50 mg/kg + PTZ exhibited a significant increase in total arm entries and spontaneous alternation compared to the PTZ model group (****p < 0.0001). It is quite remarkable that there were no significant differences in arm entries and alternation between the FC plus PTZ at doses (25, 50 mg/kg) groups (****p < 0.0001) compared to the PTZ group. These findings suggest that treating SLNC beforehand reversed the impairment in aversive long-term memory (LTM) caused by PTZ. This indicates a promising avenue for potential therapeutic interventions targeting memory impairment and neurological disorders. (^@, #^p < 0.0001). (see Table 2).

**Table 2:** Effect of orally administered SLNC and FC (25, 50 mg/kg) plus PTZ interventions on the behavioral outcomes in both the EPM test (Total Distance (cm), Time spent in open arms (s), number of entries into open arms (%)) and Y-maze (Arm Entries, Alternations) test.

		EPM		Y-Maze Test	
Groups	**Total Distance (cm)**	**Time spent in open arms (s)**	**number of entries into open arms (%)**	**Arm Entries**	**Alternations**
Control	787.0 ± 17.70	256.3 ± 5.54	21.13 ± 2.2	14.63 ± 0.74	53.00 ± 1.51
PTZ	384.3 ± 9.50^a^	41.88 ± 2.53^a^	4.87 ± 0.83^a^	5.37 ± 1.06^a^	34.63 ± 1.68^a^
Blank + PTZ	386.0 ± 5.23	44.0 ± 1.3	4.75 ± 0.70	5.37 ± 0.74	35.63 ± 1.06
SLNC25 mg/kg + PTZ	683.6 ± 4.17^b^	191.6 ± 5.01^b^	14.25 ± 1.03^b^	12.13 ± 0.99^b^	47.38 ± 1.59^b^
SLNC50 mg/kg + PTZ	701 ± 5.91^b^	197.8 ± 4.26^b^	15.38 ± 1.50^b^	12.75 ± 0.88^b^	49.88 ± 0.83^b^
FC25 mg/kg + PTZ	390.0 ± 6.59	45.63 ± 1.92	6.12 ± 1.12	5.50 ± 0.75	30.63 ± 1.06
FC50 mg/kg + PTZ	406.1 ± 9.46	51.25 ± 3.1	7.50 ± 0.92	6.00 ± 1.30	33.50 ± 0.92

Note.

a P < 0.0001 compared with the control group.

b P < 0.0001 as compared with the PTZ group alone. Each value is expressed as mean ± standard deviation (SD); n = 8 animals per group.

### 3.5 EPM test

The pretreatment SLNC plus PTZ at concentrations of 25 and 50 mg/kg groups demonstrated a notable significant difference in the total distance traveled, time spent, and number of entries into the open arms compared to the PTZ group alone (****p < 0.0001) during the 5-min test. One-way ANOVA revealed that pretreatment with FC at doses of 25 and 50 mg/kg + PTZ did not cause a significant change in the number of animal entries and time spent in the open arms compared to the PTZ group. Furthermore, the findings revealed a substantial reduction in the percentage of animal entries into the open arms, time spent, and total distance traveled by the PTZ alone group compared to the control group. (^@, #^p < 0.0001) (see Table 2).

### 3.6 OFT test

In the OFT (Fig. 2A and B), the distance moved in the center is determined to be inversely related to the level of anxiety and emotionality in the epileptic model. The OFT results showed that the number of total crossing zone centers and the average speed in the entire area in the PTZ group alone show a significant decrease compared to the control group (****p < 0.0001). The oral administration of SLNC (25,50 mg/kg) plus PTZ shows a significant increase in the average speed in the entire region and number of total crossing zone centers compared to the PTZ group alone (p < 0.0001). No significant difference was found between the groups of FC (25 mg/kg) combined with PTZ compared to the group of PTZ alone in the number of total crossing zone centers. Also, a significant difference was observed between the FC (50 mg/ml) plus PTZ group compared to the PTZ alone group for the mean speed results in the whole area (*p < 0.05). (****p < 0.0001, *p < 0.05), (Fig. 2A and B).

**Fig. 2:** The effect of SLNC and FC (25, 50 mg/kg) plus PTZ on the behavior of rats (number of total crossing zone centers (A) and average speed (B)) in the OFT test. One-way ANOVA was employed for statistical analysis. Mean ± standard deviation (SD). (****p < 0.0001, *p < 0.05).

### 3.7 Effect of SLNC and FC treatment on NO and CAT levels in the brain tissue

The data show a significant decrease in the level of CAT activity in the brain tissue of the PTZ group alone compared to the control group (****p < 0.0001). In addition, a significant increase was observed in the groups receiving SLNC (50, 25 mg/kg) + PTZ and FC (50 mg/kg) + PTZ compared to the PTZ alone group (****p < 0.0001, p ** < 0.01). (see Fig. 3). While in the group receiving FC plus PTZ, no significant change in CAT level was observed compared to the PTZ group.

**Fig. 3:** Effect of SLNC (25 and 50 mg/kg) and FC (25 and 50 mg/kg) plus PTZ on (A) CAT levels and (B) Total nitrite in brain tissue compared to the control and PTZ-injected alone groups. Mean ± standard deviation (SD); (****p < 0.0001, **p < 0.01).

In the group receiving PTZ alone, the level of NO in brain tissue was higher compared to the control group (****p < 0.0001). A significant decrease in NO levels is evident in the groups receiving SLNC (50, 25 mg/kg) + PTZ compared to the PTZ group alone (****p < 0.0001) (see Fig. 3). However, there was no significant difference between the FC (25, 50 mg/kg) + PTZ groups compared to the PTZ alone group in the amount of NO in the brain tissue.

### 3.8 Effect of SLNC and FC treatment on neuronal and spine density loss in the development of epileptic seizures

The percentage of neurons and the number of spines in the PTZ group alone decreased significantly compared to the control group (****p < 0.0001). However, there was no significant difference in the groups receiving FC (25, 50 mg/kg) plus PTZ compared to the PTZ alone group, especially in the percentage of neurons and the number of dendritic spines. On the other hand, the number of neurons and spine densities in all animals treated with SLNC (25, 50 mg/kg) plus PTZ showed a significant increase compared to the PTZ alone group. (****p < 0.0001, ***p < 0.001). (see Fig. 4).

**Fig. 4:** Effect of FC and SLNC on brain damage induced by PTZ: A representative image shows the histological examination results of brain tissue stained with Golgi, emphasizing variations in neuron count and spine density between groups. The SLNC plus PTZ groups displayed notable neuroprotection with an increased neuron count and enhanced spine density compared to PTZ alone, indicating significant preservation against PTZ-induced damage. Conversely, the FC plus PTZ groups exhibited decreased neuronal loss and spine alterations, suggesting a potential increase in PTZ's impact on brain tissue. These observations underscore the contrasting effects of FC and SLNC in minimizing brain damage. (****p < 0.0001, ***p < 0.001).

### 3.9 Immunohistochemistry of NF-κB in brain tissue

Fig. 5 shows the variation in NF-κB expression in the brain tissue of all rat groups by IHC examination. The PTZ-treated group had a significantly higher NF-κB expression than the control group (****p < 0.0001). Similarly, in the brain tissue, it is revealed that the rats receiving SLNC (25, 50 mg/kg) plus PTZ showed a notable diminish in NF-κB expression compared to the PTZ-treated (****p < 0.0001). In contrast, there was no meaningful difference between FC (25, 50 mg/kg) plus PTZ NF-κB expression compared to the group receiving PTZ alone group. (see Fig. 5) (see Fig. 6).

**Fig. 5:** Effect of orally administered SLNC and FC + PTZ on NF-κB expressions in the brain tissue against PTZ-induced stress damage. We used IHC staining to determine the level of NF-κB expressions in the brain. IHC staining images at 400× magnification. Scale bar = 80 μm. The neurons exhibit a positive brownish reaction (black arrows). (****p < 0.0001).

**Fig. 6:** Schematic representation of the study's arranged schedule for giving SLNC, FC (orally), and PTZ. It also outlines the timing for the behavior tests and examining tissues and chemicals.

## 4 Discussion

The pharmacological induction of convulsions, particularly with PTZ, is a simple technique used to trigger seizures that is used to recognize the molecular and cellular mechanisms and assess the effectiveness of AEDs [3]. PTZ-induced seizures produce a wide range of phenotypes at the neurocognitive, neurochemical, and neurophysiological [24]. PTZ hinders the function of inhibitory synapses, resulting in heightened neuronal activity. This regulation leads to seizures in animals and alters the biochemistry of the rat brain, exposing connections between neurotransmitter metabolism following seizures, energy production, protein acylation, and enzyme functions. These findings reveal a complex interplay between PTZ exposure, neurological responses, and biochemical pathways. The implications extend beyond seizure induction, suggesting broader significance for the integrity and functionality of neural networks. Understanding these complex relationships is crucial for understanding the events that occur after heightened neuronal excitation and lays the groundwork for investigating potential therapeutic interventions targeting these mechanisms [24,25]. This study aimed to examine how SLNC and FC can be neuroprotective against the severity of seizures and memory impairment caused by PTZ. Our study results indicated that administering SLNC for 4 weeks plus PTZ decreased seizure severity and improved behavioral and cognitive deficits. Most drugs cannot penetrate the BBB and, therefore, cannot impact neurons. It is crucial to comprehensively and systematically assess nano-antioxidants' effects, particularly in preventing or reducing CNS damage. These findings show that the use of nanotechnology to pass antioxidants through the BBB better and create positive changes in memory improvement may support this. Numerous studies have confirmed a clear link between the reappearance of seizures and a reduction in the number of binding sites for γ-Aminobutyric acid type A (GABAA) receptors in the hippocampus. This, in turn, leads to an increase in glutamate release and enhanced levels of NO [26,27]. Moreover, it seems that the effectiveness of monoamines on the onset of seizures is linked to their ability to regulate neuronal excitability. Lower levels of monoamines and higher nitrosative stress in animal models of epilepsy could decrease the seizure threshold, resulting in higher seizure severity scores over consecutive days [28]. The exact mechanism by which crocin exerts its anti-epileptic effects remains uncertain [29]. Previous studies have suggested a potential connection between the enhancement of the benzodiazepine receptor system and GABA [12]. However, a recent investigation conducted on rat cortical brain slices demonstrated that trans-crocetin, an active carotenoid of crocin, inhibited post-synaptic potentials in rat cingulate cortex layer I neurons, as well as depolarization induced by glutamate and N-methyl-D-aspartate. These findings reinforce the inhibitory nature of crocin and offer further insight into its potential as a treatment for epilepsy [30]. The results of our experiment show that crocin, as a bioactive compound, indicates its potential to reduce the severity of epileptic seizures by increasing CAT activity and reducing NO levels in brain tissue. Additionally, pretreatment with SLNC showed a dose-dependent reduction in seizure severity scores. It has been observed that the increase in NO levels after PTZ-induced seizures could be due to the overexpression of iNOS, an enzyme responsible for regulating NO formation. The excessive generatrion of NO can combine with O2--, resulting in the creation of peroxynitrite (ONOO-), which is known to cause harmful neurological effects [31]. Our findings are further supported by a process where crocin has been found to reduce lipid peroxidation, inhibit NO, and enhance various elements of the cell's antioxidant defenses. These abilities are believed to be linked to crocin's ability to neutralize free radicals through scavenging. Stress-associated molecular patterns (SAMPs) play a crucial role in suppressing inflammatory reactions and initiating mechanisms to maintain cellular balance [32].

Seizure development is significantly influenced by oxidative damage. Studies using animal models (in vivo) have determined that a reduction in cellular antioxidant defenses can exacerbate epilepsy in certain areas of the brain [33].

Research has shown that administering PTZ can effectively boost lipid oxidation, leading to increased levels of malondialdehyde (MDA) while decreasing important antioxidant defense mechanisms like glutathione peroxidase (GPX), CAT, and superoxide dismutase (SOD). Moreover, the absence or improper functioning of CAT, a vital antioxidant enzyme responsible for converting hydrogen peroxide into water and oxygen, appears to be associated with neurological conditions [34]. Our study revealed that PTZ can reduce the brain tissue activity of CAT. However, we discovered that SLNC pretreatment modulates these effects. Interestingly, a study conducted by Savall et al. yielded similar results. They found that the antioxidant characteristics of nanoencapsulated curcumin are the reason behind these effects. This is due to its prolonged and sustained action, which is achieved through nanoformulation [35]. In the present study, we have accomplished the successful loading of crocin onto lipid-based nanoparticles (SLNs) using an evaporation technique for synthesis. These SLNs possess a small size, which holds great promise in the treatment of neurodegenerative diseases related to the brain. SLNs have demonstrated their effectiveness as a drug delivery system, particularly in facilitating the transportation of drugs with low lipophilicity and hydrophilicity across the BBB. By incorporating these drugs into SLNs, we can significantly enhance their capability to penetrate the BBB and improve their therapeutic effects [13]. Furthermore, de Carvalho et al. [36] demonstrated that the encapsulated form of curcumin is more powerful than the non-encapsulated form in suppressing angiogenesis in a chick embryo model. The reason behind this superiority is the controlled release and enhanced absorption of the bioactive components, along with the surfactant characteristics of the polysorbate 80 (P80) coating on the nanocapsule. These factors greatly boost its capacity to penetrate cell membranes. In addition, our research group emphasized the superior effectiveness of SLNC compared to free crocin in safeguarding against oxidative damage and alleviating cognitive-like behaviors induced by PTZ administration in animals. The incorporation of crocin as a bioactive element in saffron has resulted in a significant reduction in acetylcholinesterase activity and an enhancement in serotonin levels in the nervous system [37]. These remarkable results suggest that crocin may have the capacity to enhance learning and memory in kindling-induced mice. Furthermore, research has shown that this bioactive compound can alleviate memory problems and acute damage caused by seizures in animals by protecting against oxidative damage [38,39].

In the current study, PTZ injection led to cognitive impairment in EPM and Y-maze tests by increasing anxiety and decreasing spontaneous alternations. We found that when we gave SLNC at concentrations of 25 and 50 mg/kg along with PTZ, anxiety levels decreased and the percentage of spontaneous alternations increased. The results are in line with Prathipati et al.'s research, indicating that administering curcumin-SLN has the potential to enhance cognitive function in cases of homocysteine (HCY) -induced dementia [40]. The cognitive-enhancing effects of SLNC were conducted through the OFT. The results of the OFT showed that rats pretreated with SLNC plus PTZ exhibited the ability to explore more in terms of an increase in total crossing zone centers and average speed, compared to animals treated with PC group. These findings indicate that SLNC may have potential benefits for improving cognitive performance and decreasing anxiety-like symptoms. Moreover, studies have revealed that PTZ-exposed rats have apparent impairments of spatial learning and memory that are associated with the hippocampus [41]. Pretreating with SLNC demonstrates a remarkable ability to effectively reverse these cognitive changes. Long-term use of saffron, along with its bioactive ingredient crocin, has displayed encouraging outcomes in enhancing memory function and addressing learning disabilities caused by oxidative stress and prolonged hypoperfusion in the brain [42]. Our findings not only support these studies but also emphasize that SLNC can significantly improve memory in epilepsy models. Additionally, the PTZ injection into rats resulted in notable damage to brain tissue at a histological level. The potential of crocin to mitigate the occurrence of neuroinflammation and oxidative damage may decrease the various histological changes observed in the brain, such as necrotic and degenerative alterations [30]. Utilizing crocin-loaded nanoparticles improved the overall histological integrity of the brain tissue. The IHC findings were more remarkable in the SLNC group combined with PTZ, compared to the PTZ alone group, in reducing NF-κB expression. Research has verified the potential of crocin as an NF-κB inhibitor, which ultimately suppresses cytokines. NF-κB acts as a crucial master regulator in cytokine production [30]. Excessive oxidative injury activates redox-sensitive transcription factor NF-κB due to an imbalance in reactive oxygen species (ROS) generation. While initially dormant in the cytoplasm, NF-κB becomes active and migrates to the nucleus, regulating the process of transcription. This activation triggers the increase of genes linked to inflammation and apoptosis, especially those responsible for producing inflammatory proteins in neurons [43]. NF-κB expression has been found to increase in a chronic PTZ model [44], and the interaction of crocetin, an active carotenoid of crocin, with the cellular NF-κB pathway has been reported. Additionally, crocetin treatment in mice led to a reduction in oxidative stress-mediated retinal damage in response to ischemia/reperfusion, believed to be attributed to decreased phosphorylation of NF-κB and other proteins [45]. The findings suggest that how NF-κB binding sites are arranged in DNA affects specific phosphorylation impacts. Phosphorylation at specific locations controls NF-κB's behavior. One key NF-κB subunit, p65, gets phosphorylated at many spots, influencing its functions and interactions. Notably, phosphorylating p65 at Ser536 in the transactivation area is vital for NF-κB activation. Moreover, inhibitors of nuclear factor kappa B (IκB) proteins, which block NF-κB, break down when phosphorylated, enabling NF-κB to translocate to the nucleus and bind to DNA [46]. Therefore, we can assume that SLNC treatment reduced NO/ROS generation, inhibiting PTZ-induced seizures. As a result, NF-κB activation is inhibited, protecting neurons from damage and ultimately improving cognitive abilities. Nervous system disorders frequently exhibit observable variations in dendritic spine quantity and structure. Seizures trigger a swift surge followed by a decline of dendritic spines. Chronic epilepsy models, however, have revealed a significantly more alarming pattern. They provide undeniable evidence of long-lasting damage that causes notable changes in the structure and number of dendritic spines [47]. Through the implementation of Golgi-Cox staining, the findings of this study unveiled that prior treatment with SLNC leads to a remarkable increase in dendritic spine improvement and an enhancement in the number of neurons within the cortex of animals subjected to PTZ. Multiple studies provide strong evidence for the neuroprotective effects of crocin. For example, Hassani et al. have indicated that the controlled use of crocin can result in significant antidepressant effects [48]. Studies found that crocin elevates the levels of important proteins like cAMP response element binding (CREB), brain-derived neurotrophic protein (BDNF), and vascular endothelial growth factor (VEGF) in the brain [48,49]. These proteins play a critical role in promoting neurogenesis and protecting neural tissue in this region. In addition, Batarseh et al. [50] demonstrated that treatment with Crocus sativus extract not only enhances synaptic markers but also reduces inflammation. This exciting finding further reinforces the positive impact of crocin. The results further support the notion that SLNC protects against oxidative damage and cognitive decline triggered by PTZ. Nevertheless, additional research is warranted to gain a comprehensive understanding of crocin's potential molecular targets in the signaling pathways associated with PTZ-induced degenerative processes. The remarkable progress in nanomedicine has revolutionized clinical and pharmaceutical applications by enabling pharmaceutics to effectively cross the BBB without causing disruptions to intercellular connections. This breakthrough is made possible through the use of nanocarriers that are capable of efficiently traversing the phospholipid bilayer of the BBB. Furthermore, these nanocarriers, such as SLNs, can transport drugs across various biological membranes. Recent evidence suggests that this technology holds great promise in developing innovative therapies for degenerative nerve diseases, as it allows for the targeted delivery of antioxidant drugs to suppress neuroinflammation and inhibit overactive microglia [13,15,35].

## 5 Conclusion

Our research reveals significant changes in brain histopathology, cognitive impairment, and oxidative damage induced by PTZ exposure, resulting in decreased antioxidant enzyme activities. The administration of crocin in its highly bioavailable form (SLNC) successfully reversed these effects. This provides compelling evidence of SLNC's efficient delivery to the brain and establishes, for the first time, the therapeutic potential of crocin in nanomedicine for PTZ-like symptoms, including cognitive impairment, when incorporated into lipid-based NPs. Nanomedicine has revolutionized clinical and pharmaceutical procedures by enabling medications to effectively traverse the BBB without interfering with cell connections. This breakthrough is made possible using nanocarriers that can efficiently navigate the BBB. Furthermore, nanocarriers such as SLNs can transport drugs across various biological membranes. Recent research suggests that this technology holds great promise in developing novel therapies for nerve disorders, as it facilitates the targeted delivery of antioxidant drugs to mitigate neuroinflammation.

## Funding

Not applicable.

## Statement of data availability

The data used is unavailable.

## CRediT authorship contribution statement

**Cyrus Jalili:** Writing – original draft, Visualization, Investigation, Formal analysis. **Mohammadreza Gholami:** Writing – review & editing, Formal analysis. **Seyran Kakebaraei:** Writing – review & editing, Writing – original draft, Visualization, Validation, Methodology, Investigation, Formal analysis.

## Declaration of competing interest

The authors, whose names are demonstrated below, assure that they have NO affiliations with or involvement in any organization or entity with any financial interest (such as honoraria, educational grants, participation in speakers’ bureaus, membership, employment, consultancies, stock ownership, or other equity interest; and expert testimony or patent-licensing arrangements), or non-financial interest (such as personal or professional relationships, affiliations, knowledge or beliefs) in the subject matter or materials discussed in this manuscript. In addition, the authors declare that they have no known competing financial interests or personal relationships that could have appeared to influence the work reported in this paper. also, no grants, financial support, gifts, or honoraria were received from any agency or company for the research mentioned in this manuscript.
